# Noncoding RNA as Diagnostic and Prognostic Biomarkers in Cerebrovascular Disease

**DOI:** 10.1155/2022/8149701

**Published:** 2022-04-19

**Authors:** Ruiyuan Weng, Zhiwen Jiang, Yuxiang Gu

**Affiliations:** ^1^Department of Neurosurgery, Huashan Hospital, Shanghai Medical College, Fudan University, China; ^2^Neurosurgical Institute of Fudan University, China; ^3^Shanghai Clinical Medical Center of Neurosurgery, China; ^4^Shanghai Key Laboratory of Brain Function and Restoration and Neural Regeneration, China

## Abstract

Noncoding RNAs (ncRNAs), such as microRNAs, long noncoding RNAs, and circular RNAs, play an important role in the pathophysiology of cerebrovascular diseases (CVDs). They are effectively detectable in body fluids, potentially suggesting new biomarkers for the early detection and prognosis of CVDs. In this review, the physiological functions of circulating ncRNAs and their potential role as diagnostic and prognostic markers in patients with cerebrovascular diseases are discussed, especially in acute ischemic stroke, subarachnoid hemorrhage, and moyamoya disease.

## 1. Introduction

Cerebrovascular disease (CVD) is one of the leading causes of disability and mortality worldwide. Recent epidemiological studies have shown that CVD was one of the top ten leading causes of total years of life lost worldwide, especially in China that is of great severity [1, 2]. They mainly include ischemic and hemorrhagic events, but also rare diseases such as moyamoya disease.

The human genome is characterized by a number of noncoding RNAs (ncRNAs) of unknown function. The ncRNAs are involved in many cellular processes and include microRNAs (miRNAs), long noncoding RNAs (lncRNAs), circular RNAs, and transfer RNA-derived small RNAs (tsRNAs). In addition to their intracellular activity, ncRNAs are released within extracellular vesicles in the blood, which makes them potential biomarkers in different pathological conditions [3]. Several studies have reported that circulating ncRNAs could be measured both in tissues and in biological fluids, supporting their potential use as diagnostic and prognostic markers [4–8].

In this review, we discuss the physiological functions of circulating ncRNAs and their potential role as diagnostic markers, prognostic markers, and therapeutic targets in patients with cerebrovascular diseases, including acute ischemic stroke (AIS), subarachnoid hemorrhage (SAH), and moyamoya disease (MMD). Current challenges and future perspectives are also discussed.

## 2. Biogenesis and Transport of ncRNAs

A large number of studies have demonstrated that CVDs may affect the expression level of ncRNAs in body fluids. A multitude of ncRNAs have been described in body fluids, such as serum, plasma, urine, and breast milk [9]. Different techniques have been used, including RNA sequencing, microarray screening, and real-time quantitative polymerase chain reaction (RT-qPCR) [10].

Apparently, the ncRNAs existing in body fluids mostly come from specific cells, tissues, or organs, which are quite relevant to the disease conditions, whereas there are only a few studies that provided potential mechanisms involving ncRNAs in some disease conditions. So far, five transport mechanisms of ncRNA have been described (Figure 1): (1) exosomes, (2) microparticles, (3) apoptotic bodies, (4) ribonucleoproteins, including argonaute-2 (AGO2), nucleophosmin-1 (NPM1), and high-density lipoproteins (HDLs), and (5) direct cellular connections, such as gap junctions, synapses, and intercellular bridges [10–16]. After secretion to the extracellular space, ncRNAs target specific cells and organs and exercise certain functions. Extracellular vesicles, like exosomes, microparticles, and apoptotic bodies, can transfer cargos from parental cells to recipient cells, achieving cell-to-cell communication, whereas the exact process how these extracellular vesicles are able to recognize the target cells remains unknown [10]. Ribonucleoproteins are other important carriers of ncRNAs. More than 90% of circulating miRNAs transfer through this pathway [10, 17]. The ncRNAs are quite stable and protected from RNases in body fluids, indicating that they are promising biomarkers in assessing the pathophysiological changes in the body. However, further studies are required to clarify the relationship between circulating ncRNAs and their carriers, how they interact with target cells, and what functions they exert [18].

## 3. ncRNA in Acute Ischemic Stroke

Effective management of patients with acute cerebrovascular disease relies on precise diagnosis and timely treatment, especially those with acute ischemic stroke (AIS). AIS accounts for around 80% of strokes and only has a narrow therapeutic window [19]. However, the accurate diagnosis of AIS can be disturbed by stroke mimics and other types of strokes. A computed tomography (CT) scan is usually able to detect a stroke from a blood clot or bleeding within the brain, but around half of patients are false negatives [20, 21]. MR diffusion-weighted imaging (DWI) is highly sensitive in detecting and localizing acute ischemic brain lesions but is limited by the length of the procedure, the lack of availability in remote areas, expensive costs, and prehospital settings [22]. Blood-based biomarkers with high sensitivity and specificity are therefore attractive, but those available to date have poor diagnostic accuracy [23].

Several questions in AIS diagnosis and treatment that remain to be solved can be briefly concluded as follows: the first is how to diagnose the AIS with high effectiveness and precision, which means that physicians should not only identify AIS immediately but also exclude other differential diagnoses like ICH, SAH, and stroke mimic confidently and further ascertain the stroke etiology (TOAST type) to instruct therapeutic strategies. In this setting, highly sensitive and specific biomarkers are needed in clinical practice. The second one is how to evaluate the short-term and long-term outcomes after stroke, which can be beneficial for planning subsequent therapeutic strategies and decide whether an aggressive treatment is helpful to promote poststroke recovery. To answer these questions, various investigations that focus on the ncRNA-based biomarkers are summarized as follows.

### 3.1. miRNAs as Diagnostic Biomarkers in AIS

Circulating miRNAs have been reported as potential diagnostic and prognostic biomarkers in several studies (Table 1). Using RNA sequencing data, miR-125a-5p, miR-125b-5p, and miR-143-3p were constructed to discriminate between AIS and transient ischemic attack (TIA) patients and healthy controls. Longitudinal analysis showed a significant increase in miR-125a-5p, miR-125b-5p, and miR-143-3p during the first 24 hours after AIS, with miR-125b-5p and miR-143-3p returning to normal levels within 48 hours after AIS, which reveals a good discrimination in the acute phase. A random forest classification model presented good performance in differentiating AIS and healthy controls [24]. Another study showed that serum miR-15a, miR-16, and miR-17-5p significantly increased in patients with AIS compared to healthy controls [25]. Similarly, Wang et al. reported that serum miRNA-221-3p and miRNA-382-5p were downregulated in patients with AIS [26]. The downregulation of plasma miR-30a, miR-126, and let-7b was also described in patients with AIS [27].

The miRNAs are also thought to identify stroke subtypes (Table 1). As reported by Leung et al., miR-124-3p and miR-16 are potential diagnostic biomarkers between intracerebral hemorrhage (ICH) and AIS. Plasma concentration of miR-124-3p was significantly higher, whereas the concentration of miR-16 was significantly lower in patients with ICH than in AIS patients within 24 hours after the stroke onset [28]. These findings indicated that plasma miRNAs have the potential to distinguish ICH from AIS. Kalani et al. comprehensively profiled miRNAs across acute stroke subtypes through next-generation sequencing. The sequencing data were put into LASSO regression analysis to classify AIS, ICH, and subarachnoid hemorrhage (SAH) [29]. In discriminating different ischemic stroke subtypes, miRNA can also act as an effective biomarker. A total of 87 patients with AIS and 13 healthy subjects were recruited. The ROC analysis demonstrated that miR-125b, miR-125a, let-7b, and let-7e discriminate between acute stroke due to cardiac embolism and other subtypes of stroke. Besides, miR-7-2-3p and miR-1908 showed significant AUC in both large-artery atherosclerosis and lacunar infarct patients [30].

### 3.2. miRNAs as Prognostic Biomarkers in AIS

The predictive value of miRNAs in patients with AIS is shown in Table 1. Wang et al. reported that miR-29b was significantly downregulated in patients with AIS and negatively associated with National Institute of Health Stroke Scale (NIHSS) scores and stroke volume. Of note, the overexpression of miR-29b reduced the infarct volume and brain edema and infarct volume of the brain in mice [31]. In a prospective cohort study, miRNA-150-5p was negatively associated with mortality in patients with AIS within 90 days after the stroke onset [32]. Some miRNAs related to angiogenesis, including miR-126, miR-378, and miR-101, were negatively correlated with NIHSS scores, while miR-222, miR-218, and miR-206 were positively associated with NIHSS scores [33]. The exosomal miR-223 was positively associated with AIS occurrence, stroke severity, and short-term outcomes [34]. In another study conducted by Rainer et al., plasma miR-124-3p was elevated in patients with AIS who died within 3 months after hospital admission, while miR-16 was better associated with survival [35]. A high level of serum miR-132 correlated with poststroke cognitive impairment [36], while several brain-enriched miRNAs (miR-9-5p, miR-9-3p, miR-124-3p, and miR-128-3p) were elevated in patients with infarcts larger than 2 cubic meters [37]. Overall, several miRNAs are potential biomarkers associated with the prognosis of AIS.

### 3.3. Other Biomarkers in AIS

Other ncRNAs also play an important role in diagnostic and prognostic assessment of AIS (Table 1). Recently, Zuo et al. suggested that increased plasma levels of circFUNDC1, circPDS5B, and circCDC14A may be useful to diagnose AIS. In addition, an opposite trend was observed in patients with good modified Rankin Scale (mRS) scores within 7 days, suggesting their prognostic values [38]. Like other ncRNAs, lncRNAs may change in patients with AIS. In a case-control study, a large array of differentially expressed lncRNAs were detected in blood. Specifically, lncRNA NR-002332 and lncRNA AJ131606 were upregulated, while lncRNA C10 and lncRNA f57-2 were downregulated [39]. At the same time, lncRNAs in the blood were associated with clinical outcomes: the lncRNA MIAT was significantly upregulated and correlated with the NIHSS score, mRS score, serum C-reactive protein, and infarct volume [40].

### 3.4. ncRNA as a Therapeutic Target in AIS

The secondary brain injuries are common problems after AIS, such as brain edema, ischemic reperfusion injury, and hemorrhagic transformation. Recent studies have demonstrated that ncRNAs make great contribution to exacerbate or attenuate these injury processes through affecting neuroinflammation, neural apoptosis, oxidative stress, microglia activation, and excitotoxin. Besides, neuroprotective ncRNA or their mimics can serve as promising drugs for their ability to penetrate the blood-brain barrier (BBB). Therefore, ncRNA may play a crucial role in improving AIS outcomes when serving as the therapeutic target. For example, ncRNA can influence the AIS process through regulating the oxidative stress process [41]. The upregulation of miR-424 pre- and poststroke in middle cerebral artery occlusion (MCAO) mice can decrease the cerebral infarction volume and brain edema by inhibiting oxidative stress, cellular apoptosis, and microglia activation [42], while miR-106b-5p antagomir could also decrease the infarction volume and neurological deficit in rats by regulating oxidative stress after AIS [43]. Other regulation of ncRNAs can also attenuate the oxidative stress following ischemic stroke. For example, the downregulation of miR-93 and miR-182 or the upregulation of miR-23a-3p, and miR-99a protected the AIS brain [44–47]. miR-93 antagomir alleviates ischemic injury through the Nrf2/HO-1 antioxidant pathway [47]. miR-182 promoted nitric oxide (NO) and 3-nitrotyrosine (3-NT) production and caspase-3 expression, while reducing superoxide dismutase (SOD) and manganese SOD (MnSOD) activities [46]. On the contrary, miR-23a-3p attenuated oxidative stress injury by reducing the production of NO and 3-NT and increasing the production of SOD and MnSOD [44]. All these researches indicated that miRNA might be a promising therapeutic target by attenuating the oxidative stress process.

Other miRNAs, such as miR-223 [48], miR-29b [49], miR-29c [50], miR-17-92 [51], miR-124 [52], miR-210 [53], miR-139-5p [54], miR-let-7c-5p [55], miR-107 [56], miR-207 [57], miR-335 [58], miR-22 [59], miR-9 [60], miR-378 [61], miR-122 [62], miR-210 [63], miR-455 [64], and miR-363 [65], can also reduce infarction volume and improve outcomes in animal models through various mechanisms. For example, miR-223 lowered the levels of glutamate receptors to reduce excitotoxicity and has a therapeutic role after stroke [48]. miR-139-5p agomir reduced neural apoptosis by inhibiting human growth transformation-dependent protein (HGTD-P), providing a new therapeutic insight [54].

On the contrary, the overexpression of miR-145 [66], miR-320a [67], miR-497 [68], miR-let-7f [69], miR-181a [70], miR-181b [71], miR-103-1 [72], miR-30a [73], miR-124 [74], miR-134 [75], miR-200c [76], miR-155 [77], miR-24 [78], miR-182 [46], miR-493 [79], miR-383 [80], miR-106b-5p [43], miR-15a/16-1 [81], miR-30d-5p [82], miR-337 [83], and miR-337-3p [84] exacerbates the infarction volumes, edema, and neuroinflammation. For instance, inhibition of miR-377 decreased cerebral infarct volume and suppressed cerebral inflammation but promoted angiogenesis in MCAO rats [83]. Reducing poststroke miR-200c was also a potential target to mitigate infarction volume and neurological deficit by inducing reelin expression in mice [76].

## 4. ncRNAs in Aneurysmal Subarachnoid Hemorrhage

Subarachnoid hemorrhage (SAH) is a medical emergency, accounting for 2~7% of all stroke cases, mostly due to aneurysm rupture in over 80% of cases [85]. The diagnosis of SAH mainly relies on CT scan. If the CT scan is not definitive, the next recommended diagnostic tool is the lumbar puncture [86]. Besides, SAH is also a life-threatening disease with a case fatality of 25~35%, most of which results from the subsequent cerebral vasospasm (CVS) and delayed cerebral infarction (DCI) who survive at the first bleeding event [85–89]. Therefore, the development of a predictive biomarker would be helpful to prevent the development of CVS and understand the precise mechanism behind CVS. The emerging ncRNAs suggest future developments in the diagnostic and prognostic assessment of SAH.

### 4.1. ncRNAs as Diagnostic Biomarkers in SAH

Several studies have demonstrated that the ncRNA signature in SAH was quite different from that without SAH (Table 2). A microarray analysis and RT-qPCR were utilized to confirm the association among health controls, SAH with DCI, and SAH without DCI. This single study demonstrated that serum miR-132 and miR-324 were upregulated in SAH, compared with healthy controls, while the differences between DCI and non-DCI were not statistically significant. A possible reason was that the sample size was insufficient [90]. Using a similar methodology, Lai et al. reported that miR-502-5p, miR-1297, and miR-4320 were overexpressed in patients with SAH. Seven days after diagnosis, serum miR-502-5p and miR-1297 were significantly higher in patients with SAH. Additionally, at the 7th day after SAH, serum miR-502-5p and miR-1297 levels were significantly higher in patients with increased higher World Federation of Neurological Surgeons (WFNS) and mRS at the ninth month after stroke, which can represent the worse progression of SAH [91]. Another research also determined that serum miR-1297 was directly associated with a higher WFNS grade, Hunt-Hess grade, higher Fisher score, and poor one-year outcome [92]. In cerebrospinal fluid, miR-92a and let-7b decreased, whereas miR-491 increased over time in patients with SAH [93].

### 4.2. ncRNAs as Prognostic Biomarkers in SAH

With the help of the differential expression profile of ncRNA in SAH patients' body fluids, ncRNAs are simultaneously competent to distinguish or predict some severe complications after SAH (Table 2). Stylli et al. reported that miR-27a-3p, miR-516a-5p, miR-566, and miR-1197 were expressed in cerebrospinal fluid (CSF) differently between patients with cerebral vasospasm (CVS) and those without [94]. In another study, Lu et al. described that 4 circulating miRNAs (miR-4532, miR-4463, miR-1290, and miR-4793) differentiated patients with SAH with delayed cerebral infarction (DCI) from those without DCI by using a machine learning method [95]. A further prospective case-control study demonstrated that an array of miRNA profiles were overexpressed in the CSF of patients with SAH compared with healthy controls. Of interest, the angiographic CVS after SAH was associated with an increase in miR-132-3p, -19b-3p, -210-3p, -221-3p, and -484 [96]. miR-15a and Kruppel-like factor 5 (KLF5), a potent modulator of miR-15a expression, may also be involved in CVS [97]. Several lncRNAs were also investigated in patients with SAH. According to Pan et al., lncRNAs ZFAS1 and MALAT1 were significantly upregulated, whereas lncRNAs LINC00261 and LINC01619 were downregulated in patients with SAH and CVS compared with those without CVS. Moreover, two lncRNAs (MALAT1 and LINC01619) accurately predicted CVS in around 90% of cases [98].

### 4.3. ncRNA as a Therapeutic Target in SAH

Several investigations have demonstrated that regulation of ncRNA influences many pathophysiological processes after SAH, including apoptosis, autophagy, neuroinflammation, and brain edema. Therefore, ncRNAs serve as promising therapeutic targets in SAH by regulating these underlying processes. For example, circulating exosomal miR-193b-3p treatment suppressed the expression and activity of HDAC3, reducing inflammation reaction in mice after SAH [99]. Intracerebroventricular injection of miR-103-3p antagomir before SAH reduced BBB permeability and improved neurological function [100]. Additionally, by downregulating iNOS and inhibiting the NF-*κ*B signaling pathway, miR-195-5p attenuated white matter injury and SAH-induced vasospasm [101]. Extracellular vesicle derived from the mesenchymal stem cell could transfer miR-21 to neurons, promoting neuronal survival and improving cognitive function after SAH [102]. Liang et al. showed that, in a rat SAH model, lncRNA MEG3 overexpression increased cell apoptosis [103]. Besides, other studies demonstrated that the regulation of miR-26b [104], miR-706 [105], miR-206 [106], miR-675, and let-7a [107] could also affect the brain injury and outcomes after SAH. These results might provide a deeper understanding of the pathophysiological processes in brain injury after SAH, as well as potential therapeutic targets for the translational researches.

## 5. ncRNA Biomarkers in Moyamoya Disease

Moyamoya disease (MMD) is a rare, chronic, and progressive disorder of blood vessels in the brain. MMD is characterized by progressive occlusion of the internal carotid artery or its terminal branches, associated with the formation of collateral vessels at the base of the brain [108]. It is associated with vascular cognitive impairment [109, 110] and an increased risk of stroke [111, 112]. Although the diagnosis and treatment of MMD are of high standard, the efficiency still needs improvement. According to the current guidelines from Japan [113], the diagnosis requires an angiogram. The diagnosis is mainly characterized by the morphological abnormalities of cerebral arteries but not etiological or pathogenetic abnormalities [114]. Thus, diagnostic biomarkers that can reflect the disease process are eagerly awaited.

Some studies focused on ncRNAs in MMD (Table 3). In 2014, Dai et al. reported that serum miR-106b, miR-130a, miR-126, and miR-125a-3p were differentially expressed in patients with MMD compared with healthy controls [115]. Wang et al. suggested that transfer RNA-derived fragments (tRFs) are associated with the disease [116]. Ma et al. profiled the circRNA transcriptome of circulating neutrophils in asymptomatic patients with MMD, showing a differential expression of hsa-circRNA-100146, hsa-circRNA-102534, hsa-circRNA-036592, hsa-circRNA-405463, and hsa-circRNA-405324 [117]. Similar methods have been implemented also in the whole blood of patients with MMD [118]. Another study investigated exosome miRNAs from CSF samples of 31 patients and 31 health controls, showing that miR-3679-5p, miR-6165, miR-6760-5p, and miR-574-5p had significant diagnostic power for discriminating between patients and healthy controls [119].

## 6. Current Challenges and Future Perspectives

Although several ncRNA biomarkers are currently rapidly developing, the use of ncRNA as effective biomarkers in the clinical settings still has to face some unavoidable challenges. Several ncRNAs have been tested as biomarkers in cerebrovascular diseases. They have achieved some success in distinguishing sick people from healthy controls, but sample size in these studies was relatively small and the ability of ncRNAs to discriminate between different disease subtypes or other similar diseases needs further study. At present, the sensitivity, specificity, and reproducibility of ncRNAs are not at their best. Furthermore, the standardization of sampling and testing specimens collected from different body fluids requires more investigation, since different blood centrifugation conditions, sample storage conditions, sequencing platforms, and ncRNA isolation kits can affect the outcomes [120–122]. Moreover, patients from real-life conditions have several comorbidities that may influence the expression of circulating ncRNAs, such as hypertension, diabetes mellitus, and cancer [123, 124]. Even different lifestyles, like smoking or dietary structures, affect the expression level of ncRNA. Of note, aspirin and statins may affect the expression level of circulating miR-126, miR-17, and miR92a, which influence the diagnosis of coronary artery disease when using miR-126 as a ncRNA-based biomarker [125, 126]. Additionally, the exact regulatory mechanisms of ncRNA and their physical functions are not clear. The analysis of confounding factors that affect ncRNA expression would be difficult.

Despite the shortcomings mentioned before, ncRNA biomarkers are still promising biomarkers in cerebrovascular diseases. The first ncRNA-based biomarker, lncRNA prostate cancer antigen 3, approved by FDA in 2012, has been routinely utilized in prostate cancer diagnosis, which stimulated the further development of ncRNA biomarkers in other diseases [127, 128]. ncRNAs are abundant and easily detectable in body fluids and are especially appealing as biomarkers because they are not prone to RNase degradation and remain stable in stored samples [129–131].

With the rapid development of artificial intelligence and machine learning (ML), we have never been closer to help physicians making data-driven medical decisions. The concentration of circulating ncRNAs may become essential to diagnose disease and predict outcomes. Several attempts have been made to determine their potential as biomarkers, using random forest algorithms, support vector machines, and LASSO [4–8, 24]. However, the significance of ncRNAs in cerebrovascular diseases remains poor. Further studies using ML are ongoing and will shed new light on the topic.

This review discusses the important researches about the present situation and the advance in diagnostic and prognostic ncRNA biomarkers of several cerebrovascular diseases. Although the researches of ncRNA in cerebrovascular disease remain at the preclinical stage, such studies gave us clues of understanding cerebrovascular pathophysiology and finally would drive us to a more accurate diagnosis and prognosis for cerebrovascular diseases. Further studies using ML are ongoing and will shed new light on the topic.

## Figures and Tables

**Figure 1:** Diagram of five transportation mechanisms that mediate the cell-to-cell communication of ncRNAs. ncRNAs can transport via extracellular vesicles, such as microparticles, exosomes, and apoptosis bodies. Moreover, ncRNAs can transport through binding ribonucleoproteins and through direct cellular connections.

**Table 1:** The studies about ncRNA as diagnostic and prognostic biomarkers in AIS patients.

Reference	Sample size	ncRNA	Platform	Sample	Findings
Long et al. [27] 2013	50 HC and 197 AIS	miR-30a, miR-126, let-7b	RT-qPCR	Plasma	miR-30a and miR-126 were significantly downregulated in AIS patients, while let-7b was downregulated in large-artery atherosclerosis but upregulated in other kinds of AIS patients
Leung et al. [28] 2014	79 AIS and 19 ICH	miR-124-3p, miR-16	RT-qPCR	Plasma	miR-124-3p was significantly upregulated in ICH patients, while miR-16 was significantly upregulated in AIS patients
Wu et al. [25] 2015	120 HC and 106 AIS	miR-15, miR-16, miR-17-5p	RT-qPCR	Serum	These 3 miRNAs were significantly upregulated in AIS patients
Wang et al. [31] 2015	58 HC and 58 AIS	miR-29b	RT-qPCR	Peripheral leukocyte	miR-29b was downregulated in AIS patients and was negatively associated with the NIHSS score and infract volume
Rainer et al. [35] 2016	51 AIS	miR-124-3p, miR-16	RT-qPCR	Plasma	Higher miR-124-3p was associated with mRS > 2 and mortality within 90 days; miR-16 was the opposite
Huang et al. [36] 2016	38 HC and 76 AIS	miR-132	RT-qPCR	Serum	miR-132 was higher in poststroke cognitive impairment
Dykstra-Aiello et al. [39] 2016	133 HC and 133 AIS	—	Microarray	Whole blood	lncRNA expression profiling changes after stroke and can change over time
Sørensen et al. [37] 2017	21 HC and 21 AIS	miR-9-5p, miR-9-3p, miR-124-3p, miR-128-3p	RNA-seq and RT-qPCR	CSF	miR-9-5p, miR-9-3p, miR-124-3p, and miR-128-3p were higher in bigger infarct size patients
Scherrer et al. [32] 2017	329 AIS	miR-150-5p	RT-qPCR	Plasma	Lower miR-150-5p was significantly associated with mortality within 90 days
Jin and Xing [33] 2017	Discovery: 10 HC and 10 AIS Validation: 110 HC and 106 AIS	miR-126, miR-378, miR-101, miR-222, miR-218, miR-206	RT-qPCR	Plasma	miR-126, miR-378, miR-101, miR-222, miR-218, and miR-206 were associated with the NIHSS score
Chen et al. [34] 2017	33 HC and 50 AIS	miR-223	RT-qPCR	Exosome	Upregulated miRNA was associated with the high NIHSS score and mRS > 2 within 90 days
Tiedt et al. [24] 2017	Discovery: 20 HC and 20 AIS Validation: 40 HC and 40 AIS Replication: 100 HC, 72 TIA, and 200 AIS	miR-125a-5p, miR-125b-5p, miR-143-5p	RNA-seq in the discovery cohort; RT-qPCR in the validation and republication cohort	Plasma	These 3 miRNAs' upregulation can identify the AIS from HC and TIA patients
Wang et al. [26] 2017	39 HC and 78 AIS	miR-221-3p, miR-382-5p	RT-qPCR	Serum	These 2 miRNAs were significantly downregulated in AIS patients
Zhu et al. [40] 2018	189 HC and 189 AIS	lncRNA MIAT	RT-qPCR	Peripheral leukocyte	Upregulated MIAT was associated with NIHSS scores, mRS, high-sensitivity C-reactive protein, and infarct volume
Gui et al. [30] 2019	Discovery: 13 HC and 87 AIS Validation: 20 HC and 89 AIS	miR-125b, miR125a, let-7b, let-7e, miR-7-2-3p, miR-1908	Microarray in the discovery cohort; RT-qPCR in the validation cohort	Serum	miRNAs were associated with the TOAST subtype
Kalani et al. [29] 2020	21 AIS, 17 SAH, and 19 ICH	—	RNA-seq	Exosome	The miRNA expression profiling can identify these 3 stroke types by LASSO
Zuo et al. [38] 2020	Discovery: 3 HC and 3 AIS Validation: 36 HC and 36 AIS Replication: 100 HC and 200 AIS	circFUNDC1, circPDS5B, circCDC14A	Microarray in the discovery cohort; RT-qPCR in the validation cohort and replication cohort	Plasma	These 3 circular RNAs can serve as diagnostic biomarkers and were positively associated with mRS within 7 days and infarct volumes

Abbreviation: AIS: acute ischemic stroke; CSF: cerebrospinal fluid; HC: health control; mRS: modified Rankin Scale; NIHSS: National Institute of Health Stroke Scale; RNA-seq: RNA sequencing; RT-qPCR: real-time quantitative polymerase chain reaction; TIA: transient ischemic attack.

**Table 2:** The studies about ncRNA as diagnostic and prognostic biomarkers in SAH patients.

Reference	Sample size	ncRNA	Platform	Sample	Findings
Su et al. [90] 2015	20 HC and 40 SAH	miR-132, miR-324	Microarray and RT-qPCR	Serum	miR-132 and miR-324 were higher in SAH patients
Powers et al. [93] 2016	8 SAH	—	NanoString array and RT-qPCR	CSF	miRNA expression pattern changed over time after SAH
Lai et al. [91] 2017	10 HC and 60 SAH	miR-502-5p, miR-1297, miR-4320	Microarray and RT-qPCR	Serum	miR-502 and miR-1297 were associated with WFNS and mRS at 9 months
Stylli et al. [94] 2017	4 HC and 20 SAH	miR-27a-3p, miR-516a-5p, miR-566, and miR-1197	NanoString array	CSF	These miRNAs were differentially expressed between SAH patients with and without CVS
Lu et al. [95] 2017	20 HC and 40 HC	miR-4532, miR-4463, miR-1290, and miR-4793	RT-qPCR	Plasma	4-miRNA characterized SAH patients with DCI
Bache et al. [96] 2017	10 HC and 27 SAH	miR-21 and miR-221	High-throughput RT-qPCR	CSF	2 miRNAs upregulated in SAH with DCI
Kikkawa et al. [97] 2017	3 HC and 8 SAH	miR-15a	Microarray and RT-qPCR	Plasma and CSF	The dysregulation of miR-15a and KLF4 after SAH may result in CVS
Sheng et al. [92] 2018	40 HC and 128 SAH	miR-1297	RT-qPCR	Serum	miR-1297 was associated with WFNS, Hun-Hess grade, and Fisher score and 1-year mRS
Pan et al. [98] 2020	Discovery: 10 HC and 20 SAH Validation: 65 SAH with and without CVS	lncRNA MALAT1, lncRNA LINC01619	RT-qPCR	CSF	These two lncRNA signatures can predict the occurrence of CVS

Abbreviation: CSF: cerebrospinal fluid; CVS: cerebral vasospasm; DCI: delayed cerebral infraction; HC: health control; mRS: modified Rankin Scale; RT-qPCR: real-time quantitative polymerase chain reaction; SAH: subarachnoid hemorrhage; WFNS: World Federation of Neurological Surgeons.

**Table 3:** The studies about ncRNA as diagnostic biomarkers in MMD patients.

Reference	Sample size	ncRNA	Platform	Sample	Findings
Dai et al. [115] 2014	10 HC and 10 MMD	miR-106b, miR-130a, miR-126, miR-125a-3p	Microarray	Serum	miR-106b, miR-130a, and miR-126 were upregulated in MMD, while miR-125a-3p was downregulated
Zhao et al. [118] 2017	5 HC and 5 MMD	hsa_circRNA_100914, hsa_circRNA_103343, hsa_circRNA_050898, hsa_circRNA_101720, hsa_circRNA_067209	Microarray and RT-qPCR	Whole blood	Several circular RNAs were differentially expressed in MMD compared with HC
Wang et al. [116] 2019	Discovery: 3 HC and 3 MMD Validation: 5 HC and 5 MMD	AS-tDR-000586, AS-tDR-000924, AS-tDR-007725, AS-tDR-011363	RNA-seq in the discovery cohort; RT-qPCR in the validation cohort	Whole blood	AS-tDR-000586, AS-tDR-007725, and AS-tDR-011363 were upregulated in MMD, while AS-tDR-000924 was downregulated
Ma et al. [117] 2019	5 HC and 5 MMD	hsa_circRNA_100146, hsa_circRNA_102534, hsa_circRNA_036592, hsa_circRNA_405463, and hsa_circRNA-405324	Microarray and RT-qPCR	Neutrophil	Several circular RNAs were differentially expressed in MMD compared with HC
Wang et al. [119] 2020	Discovery: 31 HC and 31 MMD Validation: 16 HC and 16 MMD	miR-3679-5p, miR-6165, miR-6760-5p, miR-574-5p	Microarray and RT-qPCR	CSF exosome	These 4 miRNAs can identify MMD from HC

Abbreviation: CSF: cerebrospinal fluid; HC: health control; MMD: moyamoya disease; RT-qPCR: real-time quantitative polymerase chain reaction.
